# Acute Outcomes of Cigarette Smoke and Electronic Cigarette Aerosol Inhalation in a Murine Model

**DOI:** 10.1155/2022/9938179

**Published:** 2022-09-22

**Authors:** Pamela Félix da Silva, Natália Alves de Matos, Camila de Oliveira Ramos, Thalles de Freitas Castro, Natália Pereira da Silva Araújo, Ana Beatriz Farias de Souza, Guilherme de Paula Costa, Sílvia Dantas Cangussú, André Talvani, Akinori Cardozo Nagato, Frank Silva Bezerra

**Affiliations:** ^1^Experimental Pathophysiology Laboratory (LAFEx), Biological Sciences Department (DECBI), Research Center in Biological Sciences (NUPEB), Federal University of Ouro Preto (UFOP), Brazil; ^2^Immunobiology of Inflammation Laboratory (LABIIN), Biological Sciences Department (DECBI), Research Center in Biological Sciences (NUPEB), Federal University of Ouro Preto (UFOP), Brazil; ^3^Immunopathology Laboratory and Experimental Pathology, Reproductive Biology Center (CRB), Federal University of Juiz de Fora, Minas Gerais, Brazil; ^4^Department of Physiology, Federal University of Juiz de Fora, Minas Gerais, Brazil

## Abstract

Cigarette smoking throughout life causes serious health issues in the lungs. The electronic cigarette (E-Cig) use increased, since it was first introduced in the world. This research work compared the short-term exposure consequences to e-cigarette vapor and cigarette smoke in male mice. Forty-five C57BL/6 mice were randomized into control (C) in an ambient air exposition cigarette smoke (CS) and aerosol electronic cigarette (EC), both were exposed to 120 puffs, 3 times/day during five days. Then, in the experimental protocol, the euthanized mice had their tissues removed for analysis. Our study showed that CS and EC resulted in higher cell influx into the airways, and an increase in macrophage counts in CS (209.25 ± 7.41) and EC (220.32 ± 8.15) when compared to C (108.40 ± 4.49) (*p* < 0.0001). The CS (1.92 ± 0.23) displayed a higher pulmonary lipid peroxidation as opposed to C (0.93 ± 0.06) and EC (1.23 ± 0.17) (*p* < 0.05). The EC (282.30 ± 25.68) and CS (368.50 ± 38.05) promoted increased levels of interleukin 17 when compared to C (177.20 ± 10.49) (*p* < 0.05). The EC developed shifts in lung histoarchitecture, characterized by a higher volume density in the alveolar air space (60.21; 55.00-65.83) related to C (51.25; 18.75-68.75) and CS (50.26; 43.75-62.08) (p =0.002). The EC (185.6 ± 9.01) presented a higher respiratory rate related to CS (133.6 ± 10.2) (*p* < 0.002). Therefore, our findings demonstrated that the short-term exposure to e-cig promoted more acute inflammation comparing to cigarette smoke in the ventilatory parameters of the animals.

## 1. Introduction

Tobacco and electronic smoking are a public health issue and a leading cause of death; thus, it is estimated that about 6 million people die worldwide each year from smoking; therefore, the mortality from smoking is expected to rise to 8 million people by 2030 [1]. Tobacco is consumed in a variety of ways, including regular cigarette, electronic cigarette (e-cig), cigar, and waterpipe, among others [2, 3]. Usually, or in general, the tobacco consumption is mainly performed with cigarettes. The burning cigarettes generate cigarette smoke (CS) and this is a complex blend, which contains more than 4500 chemical substances including carcinogens, toxins, and oxidizing compounds such as benzo-*α*-pyrenes, acrolein, carbon monoxide, nicotine, acetone, and ammonia [4]. Cigarette smoke induces the airways and lung parenchyma to elevated concentrations of reactive species; a single cigarette smoke puff contains 10^15^ to 10^17^ free radicals [4]. Regarding the elevated concentrations of reactive oxygen species (ROS), cigarette smoke depletes the antioxidant defenses [5], promoting a higher level of oxidative damage both in the short [6] and long exposition to CS [7]. In addition to inducing redox imbalance, smoking causes a higher inflammatory cell influx to the lung, mainly, macrophages and neutrophils [8]. CS activates a signaling cascade mediated by nuclear factor kappa B (NF-*κ*B) [8]; hence, this process stimulates cytokine production, proteases, and reactive oxygen species, and together, these current biomarkers increase inflammation and redox imbalance [9]. Combined, this process is a trigger for the pathophysiology of the chronic obstructive pulmonary disease (COPD) [9].

Considering that smoking is a great cause of mortality and comorbidity, strategies of cessation and prevention may improve this public health issue [10]. In this context, E-Cig are apparatuses capable of spraying a solution containing nicotine, without exposing individuals to the high content level of toxic components generated by burning tobacco [11]. The tobacco companies began introducing E-Cig as an attempt to control or lessen smoking, which has been attracting a growing number of users from all around the world [12]. In 2020, about 4.4% of adults in the United States reported using electronic nicotine delivery systems [11]. In the National Youth Tobacco Survey 2020, about 19.6% of students in high school and 4.7% of middle school students reported recurrent E-Cig usage [13].

The aerosol of electronic cigarettes contains propylene glycol, glycerin, and flavorings, as well as aldehydes and heavy metals such as nickel, copper, and other substances [14]. Once aerosolized, the compounds in the liquid go through chemical reactions, thus forming new ingredients not previously found such as carbonyl compounds [15]. In spite of being introduced as a safer form of smoking, recent results do not support the claims of decreased health risks. In animal models, exposure to E-Cig vapor is associated with cardiac inflammation and oxidative stress [16], exacerbation of the asthma inflammatory response [17], altered breast milk composition, and also the biochemical and hormonal profile in dams and offspring [18] in addition to impaired memory [19]. In humans, studies show that E-Cig vapor induces inflammation, increased risk of coughing and wheezing, promoting asthma exacerbation, as well as suppression of host defenses [20, 21]. Moreover, acute eosinophilic and lipoid pneumonia clinic manifestations have been related to E-Cig use [22]. Recently, vaping-induced lung injury cases were published, and this is a clinical condition characterized by acute and subacute lung injury, airway collapse, fluid accumulation, diffuse alveolar damage, interlobular septal thickening, and fibrosis [23]. Therefore, the focus of this study was to compare the effects of short-term exposure to EC vapor and CS in the adult mice.

## 2. Methods

### 2.1. Animals

Forty-five adult male mice (11-12 weeks old) were housed in standard laboratory cages (Laboratory of Experimental Nutrition, at UFOP, in Brazil) and had *ad libitum* access to water and food. The animals were separated into three groups (*n* =15 per group): control (C) ambient air exposition; 120 puffs/day of CS. This study had animals who were approved by Ethics Committee from UFOP (#2015/09).

### 2.2. Cigarette Smoke and Electronic Cigarette Vapor Exposure

The mice were subject to a whole-body exposure and the *in vivo* exposure systems were performed with a fixed number of puffs (120 puffs/day). In the first smoking chamber, the mice in the CS (*n* =15) were exposed to 6 commercial full-flavor filtered Virginia cigarettes, 40 puffs per exposure, corresponding to 120 puffs/day, for five consecutive days, according to the method described by Campos et al. [24].

In the second inhalation chamber, EC (*n* =15) were exposed to 120 puffs/day by electronic cigarette aerosol, divided into 3 separate times (morning, afternoon, and evening/40 puffs per exposure) during five consecutive days. The E-Cig exposures were generated from Blu-brand (Blu®, Charlotte, North Carolina, USA) disposables with nicotine (24 mg per cartridge) and purchased from a retail source. This protocol was adapted from Campos et al. [24].

The animals were placed in their respective exposure (40 cm/length, 30 cm/width, and 25 cm/height, 30 L) inside an exhaustion chapel. The cigarette or the e-cig was each attached to a 60-mL syringe at separate times, where the CS or aerosol from the EC was injected inside the inhaling chamber. The Carboxyhemoglobin (COHb) levels (%) were measured, the level of COHb in CS had a range between 0.53% and 1.97%, and EC had a range between 0.43% and 0.70%, while C ranged between 0.36% and 0.65%. The control animals were allocated in a different inhalation chamber and were exposed to ambient air [25, 26].

### 2.3. Ventilatory Parameters

After 24 h from the last exposure, the mice were sedated using a mixture of ketamine (100 mg/kg) and xylazine (20 mg/kg) administered intraperitoneally. The procedures for collecting ventilatory parameters were performed in regard to the methodology demonstrated by Araújo et al. [6, 27].

### 2.4. Blood Collection and Euthanasia

Ketamine (130 mg/kg) and xylazine (0.3 mg/kg) were utilized to euthanize the mice. Then, the animals were positioned in dorsal decubitus and a heparinized syringe (Monovette®, Sarstedt) was inserted into the third intercostal space for sample blood collection analyses. This was performed by PRIME +® VET gasometer device (Nova Biomedical, Waltham, Mass). Subsequently, the levels of COHb were determined [28].

### 2.5. Bronchoalveolar Lavage Fluid (BALF)

The BALF was analyzed as previously described by Campos et al. [26]. The thorax was taken apart, then the trachea was cannulated using an 18 G catheter; subsequently, the left main bronchus was clamped and the right lung was washed with 1.5 mL (3 x 500 *μ*L) of saline solution (0.9% NaCl). The total leukocytes count was performed in a Neubauer chamber. For the differential cell count in BALF, samples were centrifuged at 1000 RPM for 1 minute using cytocentrifuge (Shandon, Waltham, MA, USA) and the samples were stained using a rapid staining kit. Relative cell count was performed under an optical microscope with immersion oil. The total and differential cell counts were performed by two trained researchers [27, 29].

### 2.6. Lung Collection

After the BALF collection, the left lung was perfused with buffered formalin, the samples were processed, and the obtained slides were stained with hematoxylin and eosin solution (H&E). The slides were used for morphometric and histopathological measurements. The left lung from each mouse was removed, homogenized in phosphate buffer (pH = 7.5), and centrifuged for 10 minutes at 10000 RPM. The supernatant was collected and stored in freezer -80°C to perform the analyses of inflammatory biomarkers and oxidative stress markers [26].

### 2.7. Morphometric Analyses

The H&E-stained slides were used for stereological and morphometric analyses. The photomicrographs were obtained using a microscope equipped with a digital camera (Carl Zeiss AG, Oberkochen, Germany) coupled with capture software. Photomicrographs were taken using a 40x microscope objective. Twenty images from each animal were randomly obtained, and the presence and intensity of the following lesions were evaluated in a semi-quantitative manner: septal thickening, alveolar expansion, hyperemia/capillary congestion, pneumonitis, atelectasis, septal destruction, anthracosis, hemosiderosis, edema, and hemorrhage. Lesions present were classified as absent, mild, moderate, and intense, as described by de Castro et al. [30].

In regard to the semi-quantitative analysis, the volume density of the alveolar septa (Vv [sa]) and the volume density of the alveolar air space (Vv [a]) were evaluated. The analysis entailed the use of a testing system composed of 16 points and a familiar area reported by Mandarim-de-Lacerda [31].

### 2.8. Inflammatory Biomarkers on Pulmonary Parenchyma

The levels of tumor necrosis factor alpha (TNF-*α*), interleukin 17 (IL-17), and chemokine ligand 5 (CCL5) were determined in the lung parenchyma by the ELISA method. Immunoassays were performed using industrial kits from Peprotech (Ribeirão Preto, Brazil), according to the procedure described previously by Penitente et al. and Ramos *et al.* [32, 33].

### 2.9. Redox Status in Lung Homogenates

The levels of lipid peroxidation (TBARS) were determined according to the method described by Buege and Aust [34], in which, the oxidized lipid reacts with thiobarbituric acid and can be read on a spectrophotometer at 535 nm. The protein oxidation was determined according to the method described by Reznick and Packer [35]. Catalase (CAT) activity was measured from the decrease rate of hydrogen peroxide at 240 nm [36]. Superoxide dismutase (SOD) activity was measured according to the Marklund method [37], which is based on the ability of the enzyme to inhibit the auto-oxidation of pyrogallol. Total protein analysis was performed by the Bradford method [38].

### 2.10. Statistical Analyses

The sample sizes were calculated using BioEstat 5.3 software; a statistical power of 95% and a significance level of 5% were established in a pilot study. The variable used to calculate power was superoxide dismutase activity [39]. The data were expressed as mean ± standard error of the mean. The data normality evaluation was performed using the Kolmogorov-Smirnov test. Univariate analysis of variances (ANOVA one-way) followed by Tukey's post-test was used for the parametric data. The Kruskal-Wallis test and then Dunn's post-test were utilized for discrete data and expressed as median, minimum, and maximum values. The difference was considered significant when *p* < 0.05. All analyses were performed using GraphPad Prism software version 5.00 for Windows 7, GraphPad Software (San Diego, CA, USA).

## 3. Results

### 3.1. Ventilatory Parameters of Experimental Groups

Electronic cigarette (EC) exposition led to an increased RR (ANOVA, *p* < 0.002) when compared to CS. No significant differences were found when compared to Control (Table 1).

### 3.2. Influx of Inflammatory Cells in BALF

The inflammatory cells (ANOVA, *p* < 0.0001) were higher in CS and EC compared to C (*p* < 0.0001). Macrophage counts (ANOVA, *p* < 0.0001) were also higher in both CS and EC when compared to control (*p* < 0.0001). The neutrophil counts (ANOVA, *p* = 0.01) were higher in EC when compared to C and CS (*p* < 0.05). Finally, no difference was found between groups in regard to lymphocyte counts (Table 2).

### 3.3. Inflammation Biomarkers in the Pulmonary Parenchyma

The TNF-*α*, IL-17, and CCL5 were investigated to determine the inflammatory status of the lungs (Table 3). TNF-*α* levels (ANOVA, *p* = 0.03) increased in CS in comparison to C (*p* < 0.05), while IL-17 (ANOVA, *p* = 0.001) was higher in CS (*p* < 0.0001) and EC (*p* <0.05) compared to C. Finally, CCL5 levels were higher (ANOVA, *p* = 0.03) in EC when compared to C (*p* < 0.05) (Table 3).

### 3.4. Biochemical Analysis

The oxidative damage in the lungs was analyzed by enzyme activity and oxidative damage (Table 3). The lipid peroxidation (ANOVA, *p* = 0.004) increased in CS compared to C (*p* < 0.01) and EC (*p* < 0.05). Protein oxidation (ANOVA, *p* = 0.008) was higher in EC compared to C (*p* < 0.01). The activity of SOD (ANOVA, *p* = 0.0002) was decreased in CS compared to EC (*p* < 0.01) and C (*p* < 0.0001). The activity of CAT (ANOVA, *p* = 0.002) was higher in CS when compared to EC (*p* < 0.05) and C (*p* < 0.01) (Table 3).

### 3.5. Histopathological Analyses

The semi-quantitative evaluated the existence and severity of pulmonary injuries in every group. We observed that the C had almost completely preserved lung histology (Figure 1 and Table 4). The CS and EC resulted in changes in the lung parenchyma including alveolar septal thickening, alveolar lumen expansion, atelectasis, hyperemia, pneumonitis, and septal destruction (Figure 1 and Tables 4 and 5). These lesions ranged from mild to intense in severity (Table 5). Septal thickening, alveolar expansion, hyperemia, and pneumonitis were observed in all the groups; however, these lesions were more frequent in the animal groups exposed to CS and EC (Table 4). The septal thickening, atelectasis, hyperemia, and pneumonitis presented a distribution that varied mainly from mild to moderate in both, CS and EC (Table 5). On the other hand, alveolar expansion was more intense mainly in the group exposed to electronic cigarette (Table 5). Moreover, anthracosis, hemosiderosis, edema, and hemorrhage were not found in the mice studied (Table 4).

### 3.6. The Lung Parenchyma Analyses

The alveolar airway volume density (K-W, *p* = 0.002) was higher in EC (60.21; 55.00-65.83) compared to the C (51.25; 18.75-68.75) and CS (50.26; 43.75-62.08) (Figure 1(a)). We also observed that the alveolar septa volume density (K-W, *p* = 0.002) was lower in EC (39.79; 34.17-44.27) in comparison to C (48.55; 31.25-81.25) and CS (49.53; 37.92-56.35) (Figure 1(b)). The images from the animals that inhaled the EC vapor show the increased Vv of alveolar space and decreased Vv of alveolar septa in the lung (Figure 1).

## 4. Discussion

The habit of smoking is the greatest avoidable risk factor for developing COPD [40, 41]. The impact of smoking has been widely studied; cigarette smoking is prevalent worldwide. More recently, e-cig is becoming more popular, especially with young people [13]. The results showed an increase in the number of leukocytes and inflammatory markers.

Individuals that reported the use of e-cig products usually at the time of hospitalization are often hypoxic and meet systemic inflammation. In a recent research work by Layden et al. [42], in the beginning, recorded vital signs showed an abnormally rapid breathing (tachypnea) in 43% of the patients. We demonstrated for the first time that the animals exposed to E-Cig presented a higher RR when comparing the CS exposure to the mice. A higher RR occurs as a consequence from a short expositional period of the E-Cig, an effort to re-establish ventilatory balance.

We observed a higher influx of leukocytes and macrophages in BALF from the animals exposed to both CS and EC. Studies have reported that repeated CS exposition can promote prolonged lung inflammation related to leukocytes infiltration [24, 26]. Previously, Campos et al. observed the higher influx of leukocytes, especially macrophages into the airways starting from 2 days of cigarette smoke exposure [24]. Araujo et al. also demonstrated a greater influx of macrophages into the airways after five days of exposure to CS [6]. Our results corroborate with earlier findings and showed that exposure to CS, regardless of the time and number of cigarettes, is capable of promoting the recruitment of inflammatory cells to the airways.

Regarding the E-Cig, Garcia-Arcos et al. showed that E-Cig aerosol promoted increased cell numbers in BALF, with macrophages being the most abundant cell type [43]. Sussan et al. noticed a 58% increase of macrophages in BALF when exposed to E-Cig aerosols, but it did not show an impact of neutrophils, eosinophils, or lymphocytes infiltration in C57BL/6 mice [44]. Higham et al. [45] suggest that exposing cells to the aerosols from e-cig induced a neutrophil inflammatory response causing an increased release of metalloproteinase 9 and chemokine C-X-C motif ligand 8. In our research work, we determined that short-term exposition to e-cig led to macrophages and neutrophils influx into the BALF, raising questions about the usage security of these products once activated, since neutrophils recruited to the airways can produce mediators such as interleukin 8, ROS, and proteases as neutrophil elastase [46].

The inflammatory cell influx into the airways like neutrophils and monocytes is related to the increased production of inflammatory mediators. In our study, this reported increased levels of TNF-*α* in CS-exposed mice. TNF-*α* is a powerful pro-inflammatory cytokine, which acts by regulating cell apoptosis, cytotoxicity, and production of other cytokines [47]. This is a cytokine implicated in the inflammatory disease pathogenesis, as the COPD [48, 49]. Ramos et al. observed increased levels of TNF-*α* in the BALF in mice exposed to cigarette smoke for a short period [33]. Khabour et al. also reported higher levels of TNF-*α* in BALF and the mice lungs when subjected to waterpipe tobacco [3]. The synthesis of this cytokine is highly controlled and its expression is related to the mechanism via Nf-*κ*B [49]. Possibly, the increased levels of TNF-*α* in our study are related to the signaling pathways activation as the Nf-*κ*B pathway.

Exposure to e-cig promoted increased levels of the chemokine CCL-5. The CCL5 is a chemokine family member that mediates the immunological reaction. It is released by fibroblasts, platelets, monocytes, and macrophages as a result of inflammatory diseases, thus leading to the expression of inflammatory cytokines [50]. Higher levels in CCL5 were observed beforehand in the BALF of patients with COPD [51]. Few studies have evaluated the role of CCL-5 in the inflammatory response induced by e-cig aerosol. Pham et al. noticed that E-Cig exposure promoted increased expression of CCL-5 in a breast cancer model; however, when compared to the findings from our study, it was a difficult comparison since the response to cancer cells to a stimulus is different than that of healthier cells [52]. However, Pan et al., while evaluating the function of CCL5 in vivo, recognized that increased levels of this cytokine promoted increased neutrophil recruitment to the airways and exacerbation of asthma [53]. This is related to the results detected in our study, and it suggests that E-Cig acts by regulating CCL5 expression, and the increase in this chemokine causes the recruitment into the lungs.

Furthermore, we showed that a brief exposition to CS and EC vapor promoted in higher interleukin 17 levels. IL-17 is a cytokine originally identified as playing a main role in the defense against microorganisms [54]. Moreover, this cytokine is identified in the pulmonary biopsies of patients with COPD and in the sputum of patients during exacerbations of the disease [55], suggesting that although our model is a short exposure, the increase in IL-17 levels induced by conventional and e-cig may increase the risk of EC might elevate the risk of COPD development.

In order to evaluate the outcome of CS and EC exposure in the lung, we assessed the redox imbalance in the lung parenchyma. CS has a variety of free radicals per puff, and it is a powerful source of oxidative stress. In our previous studies, we demonstrated that exposition to CS is capable of modifying the activity of antioxidant enzymes, consequently causing oxidative injury to the cellular constituents as lipids, proteins, and DNA [24, 26]. However, the effects of exposition to EC vapor on the redox status in the lung are still uncertain.

SOD is considered the first line of enzymatic defense of an organism, as it was responsible for the dismutation of the superoxide anion in hydrogen peroxide, a substrate for the enzyme CAT. In our research work, the SOD activity decreased in the mice subjected to EC, thus suggesting that the exposure caused an increase in O_2_^–^ concentration since this enzyme has reduced activity when there is an overload of its substrate. It is also important to emphasize that nicotine is responsible for an increase in O_2_^−^ concentration through the activation of the NADPH oxidase (NOX) enzyme complex so that when it binds to nicotinic acetylcholine receptors, nicotine promotes entry of Ca^2+^ into the cells activating the protein kinase C, which in turn activates NOX, leading to oxidative stress [56]. The excess O_2_ may have been directed to the peroxynitrite pathway in a reaction that occurs three times faster than the SOD catalyzed reaction favoring lipid peroxidation [57]. Our data corroborate with Campos et al., where we observed that a brief CS exposure is associated with oxidative stress and a decrease in SOD activity [24]. Interestingly, we noticed an increased activity of CAT in the mice subjected to CS, which also revealed a raised level in the antioxidant defense system against the insults offered through E-Cig and CS.

A brief exposure to CS and e-cig induces damage to cell macromolecules. Previously, Campos et al. demonstrated elevated lipid peroxidation in animals exposed to CS [24]. Mayyas et al. observed increased levels of lipid peroxidation in the mice subjected to EC vapor [16]. In our study, we did not find any additional lipid oxidation in the E-Cig exposed group; however, increased levels of protein oxidation were measured. Our results corroborate previous findings and demonstrate that e-cig also act to promote oxidative damage.

The animals subjected to inhaled CS did not show changes in lung histoarchitecture. Therefore, we believe that the five-day exposure was not enough to produce alterations in the alveoli structure using only 6 commercial cigarettes per day. Recently, Araújo et al. showed that short-range/or shorter-term exposure using the 12 commercial cigarettes per day promoted damage to the lung parenchyma characterized by an alveolar volume density increase and an alveolar septal volume density decrease [6].

However, the E-Cig was able to induce structural change in the pulmonary architecture of C57BL/6 mice during only five days and this is the first time that any study has shown these structural changes. Lerner and collaborators [58] showed that human pulmonary fibroblasts exhibited both straining and morphological abnormalities/alterations/shifts in reaction to E-Cig in a short exposure model; moreover, after 24 hours, the fibroblasts exhibited various morphological alterations suggesting that E-Cig affects inducing a straightforward manner to the pulmonary cells that affect the morphology of the cells, thus promoting a phenotype strain and therefore contributing to the inflammative reaction in a way which depends on the nicotine concentration amount and taste preference. Our research work estimated that the EC has led to structural changes in the lungs as a consequence of the redox and inflammation response in pulmonary cells exposed to the aerosol, and also, we suggest that these shifts in lung architecture promoted by a short exposition to E-Cig reflected a modified respiration-controlled equilibrium, once we demonstrated that E-Cig showed a higher pulmonary rate in comparison to the CS.

The current study presents some limitations. Firstly, in general, we showed the inflammatory and oxidative effects; however, we believe that the mechanisms associated in the responses stimulated by the cigarettes are different; therefore, further studies are needed. Secondly, even though there are more inflammatory mediators associated with the recruitment of inflammatory cells into mice lungs. Furthermore, another potential limitation includes a unique gender used, the short duration of cigarette exposures, and the absence of a methodology for detecting the actual concentration of nicotine contained in the vapor. This research needs to be acknowledged and further investigations ought to be performed in the future.

In conclusion, these findings suggest the potential dangers in pulmonary biology associated with cigarette and E-Cig use even after a few days of exposure.

## Figures and Tables

**Figure 1:** Assessments of alveolar airspace and alveolar septa. Representative images of the lung stained with H&E. Bar =50 *μ*m, 400x augmentation. (a) Vv of alveolar airspace. (b) Vv of alveolar septa. (a) represents a significant difference in comparison to C. (b) represents a significant difference when compared to CS. Results were expressed as median (minimum and maximum) and were analyzed by the Kruskal-Wallis test followed by Dunn's post-test (*p* < 0.05, *n* =10 each group). C: control; CS: cigarette smoke; EC: electronic cigarette.

**Table 1:** Analysis of pulmonary function parameters.

	C	CS	EC	*p* value
RR (breaths/min)	163.0 ± 2.5	133.6 ± 10.2	185.6 ± 9.01^b^	*p* < 0.002
VT (mL)	0.28 ± 0.01	0.33 ± 0.05	0.35 ± 0.03	*p* = 0.41
Vmin (mL/min)	46.18 ± 1.35	45.74 ± 8.6	55.7 ± 3.8	*p* = 0.38
Body mass (g)	29.0 ± 0.9	30.2 ± 0.5	29.2 ± 0.7	*p* = 0.46

C: control; CS: cigarette smoke; EC: electronic cigarette; RR: respiratory rate; VT: tidal volume; Vmin: minute ventilation. (b) represents a difference compared to CS. Data were expressed as mean ± SEM and were analyzed by one-way ANOVA followed by Tukey's post-test (*p* < 0.05).

**Table 2:** Effects of cigarette smoke and electronic cigarette aerosol on the influx of cells in bronchoalveolar lavage.

	C	CS	EC	*p* value
Leucocytes (x10^3^/mL)	118.00 ± 5.53	220.00 ± 6.49^a^	234.00 ± 7.02^a^	*p* < 0.0001
Macrophages (x10^3^/mL)	108.40 ± 4.49	209.25 ± 7.41^a^	220.32 ± 8.15^a^	*p* < 0.0001
Lymphocytes (x10^3^/mL)	7.81 ± 2.28	8.52 ± 1.79	8.89 ± 1.74	*p* = 0.92
Neutrophils (x10^3^/mL)	1.80 ± 3.44	2.23 ± 6.67	4.79 ± 1.00^a,b^	*p* = 0.01

C: control; CS: cigarette smoke; EC: electronic cigarette. The letter (a) represents a significant difference compared to C; the letter (b) represents a significant difference compared to CS. Data were expressed as mean ± SEM and were analyzed by one-way ANOVA followed by Tukey's post-test (*p* < 0.05).

**Table 3:** Immunoenzymatic assay and biochemical evaluation on pulmonary parenchyma.

	C	CS	EC	*p* value
TNF-*α* (pg/mL)	92.86 ± 10.88	157.00 ± 21.40^a^	128.50 ± 11.24	*p* = 0.03
IL-17 (pg/mL)	177.20 ± 10.49	368.50 ± 38.05^a^	282.30 ± 25.68^a^	*p* = 0.001
CCL5 (pg/mL)	157.80 ± 10.63	264.80 ± 34.52	343.60 ± 66.58^a^	*p* = 0.03
TBARS (nmol/mg protein)	0.93 ± 0.06	1.92 ± 0.23^a,c^	1.23 ± 0.17	*p* = 0.004
Protein carbonyl (nmol/mg protein)	3.68 ± 0.47	5.71 ± 0.62	7.24 ± 0.84^a^	*p* = 0.008
SOD(U/mg protein)	120.80 ± 4.76	72.59 ± 8.84^a,c^	112.30 ± 2.82	*p* = 0.0002
CAT (U/mg protein)	2.94 ± 0.18	5.59 ± 0.48^a,c^	3.50 ± 0.56	*p* = 0.002

C: control; CS: cigarette smoke; EC: electronic cigarette. The letter (a) represents a significant difference compared to C; (c) represents a significant difference compared to EC. Data were expressed as mean ± SEM and were analyzed by one-way ANOVA followed by Tukey's post-test (*p* < 0.05).

**Table 4:** The existence of injuries in the experimental groups.

Injuries	C *n* =10 (%)	CS *n* =10 (%)	EC *n* =10 (%)
Septal thickening	3 (30.0)	8 (80.0)	6 (60.0)
Alveolar expansion	2 (20.0)	5 (50.0)	10 (100.0)
Atelectasis	0 (0.0)	6 (60.0)	3 (30.0)
Hyperemia	2 (20.0)	4 (40.0)	4 (40.0)
Pneumonitis	3 (30.0)	7 (70.0)	8 (80.0)
Destruction septal	0 (0.0)	10 (100.0)	10 (100.0)

C: control; CS: cigarette smoke; EC: electronic cigarette.

**Table 5:** Semi-quantitative analysis of lung injuries from the animals that inhaled in the CS and EC.

Injuries	None *n* (%)	Light *n* (%)	Medium *n* (%)	Severe *n* (%)	Total%
Septum thickening					
CS	2 (20)	3 (30)	4 (50)	1 (10)	100
EC	3 (30)	4 (40)	3 (30)	0 (00)	100
Alveolar expansion					
CS	5 (50)	1 (10)	3 (30)	1 (10)	100
EC	0 (00)	2 (20)	3 (30)	5 (50)	100
Atelectasis					
CS	5 (50)	3 (30)	1 (10)	1 (20)	100
EC	7 (70)	2 (20)	1 (10)	0 (00)	100
Hyperemia					
CS	6 (60)	4 (40)	0 (00)	0 (00)	100
EC	6 (60)	4 (40)	0 (00)	0 (00)	100
Pneumonitis					
CS	3 (30)	4 (40)	1 (10)	2 (20)	100
EC	2 (20)	4 (40)	4 (40)	0 (00)	100

CS: cigarette smoke; EC: electronic cigarette.

## Data Availability

The data obtained in this study are available from the corresponding author upon request.
